# Comparison of bone morphogenetic protein and autologous grafting in the treatment of limb long bone nonunion: a systematic review and meta-analysis

**DOI:** 10.1186/s13018-020-01805-4

**Published:** 2020-07-29

**Authors:** Yong-Qiang Zhou, Hong-Liang Tu, Yan-Ji Duan, Xiao Chen

**Affiliations:** 1 The Department of Orthopedic Surgery, The First People’s Hospital of Neijiang, Neijiang, 641000 Sichuan China; 2 The Department of Neonatology, The First People’s Hospital of Neijiang, Neijiang, 641000 Sichuan China

**Keywords:** Bone morphogenetic protein, Autologous bone graft, Nonunion, Long bone, Meta-analysis

## Abstract

**Background:**

Bone morphogenetic proteins (BMPs) have strong bone induction properties and can promote healing of fractures and other defects. However, BMP treatment efficacy for long bone nonunion remains controversial. The aim of this meta-analysis was to synthetically evaluate the advantages and disadvantages of BMP plus bone grafting (observation group) versus autologous bone grafting (control group) for limb long bone nonunion.

**Methods:**

PubMed, Embase, Web of Science, Cochrane Library, OVID, CNKI, Weipu Journal, Chinese Biomedical Literature, and WanFang were searched for randomized and non-randomized controlled trials published before November 2019. A meta-analysis of outcome indicators was performed using RevMan 5.3 and Stata 12.0.

**Results:**

Five randomized and four non-randomized controlled trials involving 30–124 cases were included, with a total of 655 nonunion cases. There were no significant group differences in postoperative healing rate, infection, and secondary operation rates (*P* > 0.05), but the study group demonstrated significantly shorter mean healing time (WMD = − 1.27, 95%CI − 1.67 to − 0.88, *P* < 0.00001), a greater frequency of excellent/good post-treatment limb function (RR = 1.18, 95%CI 1.01–1.39, *P* = 0.04), and lower intraoperative blood loss (*P* < 0.05). Alternatively, the hospitalization cost was significantly higher in the study group (*P* < 0.01).

**Conclusions:**

Bone morphogenetic protein is a viable alternative to autologous bone grafting, with potential advantages of accelerated fracture healing and improved postoperative function.

## Introduction

Nonunion of long bone fractures is observed in 2.5 to 46% of cases depending on the location and severity of damage to the bone, soft tissue, and vascular structures [1]. Treatment of nonunion involves mechanical fixation and biological repair, often requiring autologous bone grafting to assist in bone healing. At present, autologous bone is the only graft with the capacities for osteogenesis, bone induction, and bone conductivity, and as such is still the “gold standard” for bone graft material [1, 2]. The main source for autologous bone for grafting is the iliac crest due to its accessibility and the abundance of progenitor cells and growth factors [1, 2]. However, obtaining autologous bone frequently results in minor complications (9–39%) and occasionally severe complications (0.76–25%) [3, 4] such as infection, hematoma, chronic pain in the donor area, hernia, and residual scarring [2, 5]. In addition, the quality of autologous bone varies among individuals and age groups, limiting the clinical application [6, 7].

Developments in bone tissue engineering and bone biology have revealed the unique advantages of bone morphogenetic proteins (BMPs) for bone tissue repair. Members of the transforming growth factor superfamily, BMPs, promote bone healing by inducing mesenchymal stem cells to differentiate into osteoblasts [8, 9]. Two BMPs (recombinant BMP 2 and recombinant BMP 7) have been approved for clinical use by the US Food and Drug Administration (USDA) [10]. Healing rates as high as 92.3% have been reported in nonunion patients following surgical debridement and fixation with additional BMP treatment [11]. In fact, some clinicians believe that BMP can replace autologous bone transplantation [12, 13]. While a meta-analysis by Dai et al. [14]. concluded that BMPs have not yet surpassed autologous bone transplantation as the optimal treatment for acute tibial fractures and nonunion, the included studies were of small sample size and the subject selection was not restricted to nonunion. Therefore, we conducted a systematic review and meta-analysis of currently available studies to evaluate the advantages and disadvantages of BMP versus autologous bone grafting for the treatment of limb long bone nonunion.

## Materials and methods

### Search strategy

We searched PubMed, Embase, OVID, Web of Science, Cochrane Library, WanFang, CNKI, and CBM databases using combinations of the following keywords: “bone morphogenetic protein,” “BMP,” “osteogenic protein-1,” “autologous bone graft,” “long bone,” “nonunion,” and “randomized controlled trials” (last updated on November 30, 2019). Google Scholar was also searched to identify potentially relevant literature. In addition, reference lists of identified reports were reviewed for other potentially relevant studies. Language and publication status were not restricted, and gray literature as well as ongoing trials were also investigated. All studies were carefully evaluated for the replication of the same data. Criteria used to define duplicate data included study period, hospital, treatment information, and any additional inclusion criteria.

### Inclusion and exclusion criteria

Inclusion criteria were as follows: (1) randomized and non-randomized controlled clinical trials of BMP plus autograft for treatment of nonunion without restrictions on country of origin; (2) patients aged 18 years and older with nonunion of tibia, fibula, femur, ulna, radius, or humerus more than 6 months after fracture; (3) treatment with BMP alone or BMP combined with bone graft in the observation group and autologous bone graft in the control group; and (4) publication in English or Chinese. Exclusion criteria were as follows: (1) article type specified as “review,” “letter,” “conference report,” “case report,” or “animal study” and studies without usable data; (2) infection without control; (3) pathological fracture or congenital bone nonunion; (3) less than 6 months of follow-up, incomplete data, or errors; and (4) duplicate data from another study.

### Data extraction and quality assessment

Two authors independently extracted the data from all eligible articles, and any disagreements were resolved by discussion and consensus among the authors. Information retrieved from each study included author names, year of publication, country of origin, study design, methods, number of patients, postoperative healing rate, infection rate, secondary operation rate, frequency of excellent/good post-treatment limb function, mean healing time, operation time, intraoperative blood loss, hospitalization cost, and length of hospital stay. We also evaluated the potential for bias in all included studies. For non-randomized trials, the Newcastle-Ottawa Scale (NOS) was used for bias assessment. For randomized controlled trials, evaluation criteria and methods followed the Cochrane Collaboration proposal. Appraisal criteria included random sequence generation, allocation concealment, blinding of participants and personnel, blinding of outcome assessment, incomplete outcome data, selective reporting, and other sources of bias. Each of these factors was recorded as low risk, unclear risk, or high risk.

### Statistical analysis

#### Heterogeneity test and effect value

A meta-analysis of pooled data was conducted using the Review Manager 5.3 and Stata 12.0 software. Standardized mean differences or weighted mean differences (WMDs) were calculated for continuous variables. Risk ratios (RRs) were calculated for dichotomous variables in each study, and 95% confidence intervals (CIs) were determined for all effect sizes. Statistical heterogeneity across trials was quantified by the *I*^2^ statistic according to PRISMA guidelines. A value of *I*^2^ less than 25% was considered indicative of homogeneity, and values of 25%, 50%, and 75% or more were considered indicative of low, moderate, and high heterogeneity, respectively. For homogeneous studies or those with low statistical heterogeneity, the fixed-effects model was used to determine the overall RR or WMD. Otherwise, the random-effects model was used. Sensitivity analyses were conducted by removing each study individually to assess heterogeneity and robustness of the pooled results. Datasets causing significant changes in pooled results when removed were analyzed further to assess the reason. We then judged the results for stability and strength. If the heterogeneity was too large to analyze, descriptive analyses are presented.

#### Publication bias

We assessed potential publication bias using Begg and Egger tests. All tests were two-tailed, and a *P* < 0.05 was considered significant.

## Results

### Search results

A total of 511 publications were selected from the initial search, of which 143 were duplicates and 256 did not match our inclusion criteria according to title and abstract assessment. No data were obtained from the gray literature or ongoing trial searches (we received no answers from the authors we contacted). Of the remaining 112 studies retrieved, 103 did not meet the inclusion criteria after the full-article assessment. Finally, 5 randomized controlled trials (RCTs) [15–19] and 4 non-randomized controlled trials [20–23] were included in the systematic review and meta-analysis, most of which were small sample size studies of 30–124 cases, with a total of 655 nonunion cases. These 9 studies [15–23] reported on 11 trials as one (Hackl et al. [23]) reported 3 clinical trials. The observation group was treated with BMP plus autologous bone in 5 studies, BMP alone in 2 studies, and BMP combined with natural inorganic bone in one study. In the ninth study, the observation group consisted of 18 cases receiving BMP alone and 8 cases receiving BMP plus autologous bone grafting. All control groups received autologous bone grafts, and all patients in both groups underwent mechanical fixation (intramedullary nail, plate, screw, minimally invasive stabilization system, external fixation, etc.). The literature search and selection process are illustrated in Fig. 1.

**Fig. 1:** PRISMA flowchart of the study selection process

### Study characteristics

The primary characteristics of the 9 selected studies are summarized in Table 1. According to the Cochrane Collaboration Risk of Bias Tool, the quality of 4 RCTs was acceptable (Fig. 2). The non-randomized controlled trials were also considered to be of high quality according to the Newcastle-Ottawa Scale (Table 2).

**Table 1:** Summary of study and patient characteristics

Study	Study type	Country	Intervention	Case	Age, years	M/F	Nonunion time (months)	Follow-up (months)	Outcome
Cook [15]	RCT	USA	BMP Autologous bone	14 16	– –	23 7	27.2	> 9	(1), (2)
Chen et al. [19]	RCT	China	BMP + inorganic bone Autologous bone	20 30	35 35	– –	8.5	13.9 (8–60)	(1), (3)
Friedlaender et al. [16]	RCT	USA	BMP + autologous bone Autologous bone	63 61	38 34	88 34	17	24	(1), (2), (5)
Zimmermann et al. [20]	n-RCT	Germany	BMP + autologous bone Autologous bone	26 82	51 44	82 26	10 11	> 12	(1), (2) (5)
Tressler et al. [21]	n-RCT	USA	BMP Autologous bone	19 74	45.11 41.69	57 36	> 6	20 ± 17.7	(1), (2)
von Ruden et al. [17]	RCT	Germany	BMP + autologous bone Autologous bone	24 25	43 45	38 11	11	14 (6–8) 15 (6–54)	(1), (3)
Yin et al. [22]	n-RCT	China	BMP + autologous bone Autologous bone	26 21	38 39	35 12	–	10–24	(1), (3), (4)
Hackl et al. [23]	n-RCT	Germany	BMP + autologous bone Autologous bone	62 50	–	75 37	–	> 12	(1), (4)
Humerus				13/9	49.0/51.0	13/9	14.8 ± 3.8		
Femoral				28/13	55.2/42.4	28/13	11.7 ± 1.1		
Tibia				21/28	51.6 42.3	34/15	10.3 ± 2.6		
Liu et al. [18]	RCT	China	BMP + autologous bone Autologous bone	22 20	42.25 41.57	26 16	–	6–24	(1), (3), (4), (5)

*RCT* randomized controlled trial, *n-RCT* non-randomized controlled trial, *BMP* bone morphogenetic protein

(1) Postoperative healing rate, (2) postoperative infection rate, (3) excellent and good rate of limb function, (4) the mean healing time, (5) secondary operation rate, (6) operation time, (7) intraoperative blood loss, (8) hospital stay, and (9) the hospitalization cost

**Fig. 2:** Risk of bias summary (**a**) and assessment summary (**b**) of randomized controlled trials (green = low risk; red = high risk; yellow = unknown)

**Table 2:** Quality evaluation of non-randomized controlled trials (NOS)

Study	First item	Second item	Third item	Fourth Item	Fifth item	Sixth item	Seventh item	Eighth item	Scores
Zimmermann et al. [20]	1	1	0	1	2	1	1	1	8
Tressler et al. [21]	1	1	1	1	2	1	1	1	9
Yin et al. [22]	1	1	0	1	2	1	1	1	8
Hackl et al. [23]	1	1	0	1	2	1	1	1	8

### Results of meta-analysis

#### Postoperative healing rate

Postoperative healing rate was evaluated in nine studies [15–23]. The meta-analysis revealed no significant difference in the final healing outcome between the observation and control groups (RR = 1.00, 95%CI 0.94–1.07, *P* = 0.89, Fig. 3) with low heterogeneity among studies (*P* = 0.07, *I*^2^ = 42%). In the sensitivity analysis, removal of Zimmermann et al. [20] significantly reduced the study heterogeneity (*I*^2^ = 0%, *P* = 0.54) but had only modest effects on the pooled results (RR = 0.97, 95%CI 0.90–1.04, *P* = 0.34). Analysis of the causes of heterogeneity revealed that all cases in Zimmermann et al. (2009) had a previous history of failed autologous bone graft repair, and BMP was used as an alternative treatment. It is possible that such patients demonstrate better BMP responsiveness than patients without previous bone graft repair. There were also fewer patients in the BMP group than the control group, which may have added heterogeneity to the pooled sample.

**Fig. 3:** Forest plot of postoperative healing rate after treatment with bone morphogenetic protein (BMP) alone or plus bone grafting versus autologous bone grafting for nonunion

Five studies [16–18, 22, 23] used BMP combined with autologous bone transplantation in the observation group and autologous bone transplantation alone in the control group. There was no statistical heterogeneity among the groups (*I*^2^ = 0%, *P* = 0.42), so the fixed-effect model was adopted. The meta-analysis revealed no significant difference in the postoperative healing rate between the observation and control groups (RR = 0.99, 95%CI 0.92–1.07, *P* = 0.86, Fig. 4a). Only two studies [15, 21] used BMP alone in the observation group, but there was no significant heterogeneity so a fixed-effects model was applied (*I*^2^ = 0%, *P* = 0.48). The pooled results indicated no significant difference in 1 postoperative healing rate between the two groups (RR = 0.84, 95%CI 0.67–1.05, *P* = 0.13, Fig. 4b).

**Fig. 4:** Forest plot of postoperative healing rate after BMP combined with bone grafting (**a**) and BMP alone (**b**) versus autologous bone grafting alone for nonunion

Five studies [15, 16, 19, 20, 23] examined the nonunion of the tibia. There was no significant difference in postoperative healing rate between the observation group (BMP or BMP combined with autologous bone transplantation) and the control group (RR = 1.01, 95%CI 0.90–1.13, *P* = 0.92, Fig. 5) but with high heterogeneity between the groups (*I*^2^ = 65%, *P* = 0.02). A sensitivity analysis showed that the heterogeneity decreased substantially after excluding Zimmermann et al. [20] (*I*^2^ = 0%, *P* = 0.52), while the outcome comparison was not significantly altered (RR = 0.95, 95%CI 0.87–1.03, *P* = 0.21).

**Fig. 5:** Forest plot of postoperative healing rate after BMP or BMP combined with autologous bone versus autologous bone grafting for tibial nonunion

In conclusion, there were no significant differences in the postoperative rate between the BMP and control groups. Further, the combination of autogenous bone with BMP did not alter this result. In addition, the outcome did not differ between the groups for nonunion of any long bone and nonunion specifically in the tibia. Sensitivity analysis also showed that the results of the meta-analysis were stable.

#### Postoperative infection rate

Four studies [15, 16, 20, 21] provided data on postoperative infection rate, including 116 patients in the BMP group and 222 in the control group. There was no statistical heterogeneity (*I*^2^ = 0%, *P* = 0.83) and no significant difference in the outcome between the groups (RR = 0.96, 95%CI 0.53–1.77, *P* = 0.91, Fig. 6).

**Fig. 6:** Forest plot of postoperative infection rate after BMP or BMP combined with autologous bone versus autologous bone grafting for nonunion

#### Excellent and good rate of limb function

Postoperative excellent/good postoperative limb function rate was documented in 4 articles [17–19, 22]. A fixed-effects model was applied because no statistical heterogeneity was found (*I*^2^ = 0%, *P* = 0.68). There was a significant difference in the outcome between the observation and control group (RR = 1.18, 95%CI 1.01–1.39, *P* = 0.04, Fig. 7). The Chen et al. [19] study treated the observation group using BMP plus natural inorganic bone, which may have a disproportion influence on the outcome; however, removing this study had little effect on the pooled results (RR = 1.22, 95%CI 1.01–1.47, *P* = 0.04).

**Fig. 7:** Forest plot of excellent/good functional recovery rate after BMP combined with autologous bone versus autologous bone grafting for nonunion

#### The mean healing time

Three articles [18, 22, 23] with 201 patients reported data on the mean healing time. A fixed-effects model was applied because low heterogeneity was found among the studies (*I*^2^ = 21%, *P* = 0.28). Mean healing time was significantly shorter in the observation group compared to the control group (WMD = − 1.27, 95%CI − 1.67 to − 0.88, *P* < 0.00001, Fig. 8).

**Fig. 8:** Forest plot of mean healing time after BMP combined with autologous bone versus autologous bone grafting for nonunion

#### Secondary operation rate

Three studies [16, 18, 20] provided data on secondary operation rate with moderate heterogeneity (*I*^2^ = 56%, *P* = 0.10) and no significant difference in the outcome between the groups (RR = 0.55, 95%CI 0.19–1.64, *P* = 0.29, Fig. 9).

**Fig. 9:** Forest plot of secondary operation rate after BMP or BMP combined with autologous bone versus autologous bone grafting for nonunion

#### Operation time and intraoperative blood loss

Two articles reported the operation time and intraoperative blood loss. Descriptive analyses are presented because the BMP intervention differed between the 2 studies. In Yin et al. [22], the BMP combined with autologous bone graft group included 26 patients and the control group 21 cases. Operation time was significantly shorter in the observation group than in the control group (70.96 ± 13.34 vs. 101.67 ± 12.78 min; *P* < 0.01). Tressler et al. [21] also compared the operation time as well as the intraoperative blood loss between 19 cases receiving BMP alone and 74 cases in the control group. The operation time was again significantly shorter in the observation group compared to the control group (168.9 ± 86.5 vs. 257.9 ± 93 min, *P* < 0.01). The intraoperative blood loss was also lower in the observation group (331.6 ± 357.2 vs. 554.6 ± 447.8 mL, *P* = 0.02).

#### Hospital stay and the hospitalization cost

One study each reported the length of hospital stay and hospitalization cost. Tressler et al. [21] found a shorter hospital stay in the observation group, although the difference did not reach significance (3.2 ± 2.6 vs. 3.8 ± 2.5 days, *P* = 0.37), while Yin et al. [22] found a higher average hospitalization cost in the observation group compared to the control group (2.65 ± 0.34 vs. 2.14 ± 0.35 in units of ten thousand Yuan, *P* < 0.01).

#### Publication bias

The large sample sizes of some pooled outcomes, such as postoperative healing rate, allowed for the application of Begg’s test and Egger’s test for the analysis of publication bias. No significant bias was found across studies by either test (Begg test, *P* = 0.592, Fig. 10a; Egger test, *P* = 0.863, Fig. 10b).

**Fig. 10:** Publication bias for postoperative healing rate after BMP or BMP combined with autologous bone versus autologous bone grafting for nonunion. **a** Begg’s funnel plots. **b** Egger’s funnel plots

#### Sensitivity analysis

Sensitivity analysis indicated our current data was relatively steady and credible (Fig. 11).

**Fig. 11:** Sensitivity analysis of postoperative healing rate after BMP or BMP combined with autologous bone versus autologous bone grafting for nonunion

## Discussion

Nonunion of long bone fracture is associated with a greater risk of complications and poor long-term prognosis [24]. Numerous factors influence fracture healing, including fracture type, fracture site, degree of surgical dissection, fracture end stability, infection, poor mechanical fixation, inadequate blood supply, malnutrition, and chronic disease [6, 25]. Most fractures heal within 20 weeks, and nonunion is defined as incomplete healing within 6 months [26]. Bone repair can be induced by local biological stimulation at the fracture site when healing is delayed or nonunion occurs. At present, autologous bone grafting remains the “gold standard” [1, 2, 20, 22] by which other treatment options are compared. However, autologous bone harvesting can result in chronic pain, scarring at the donor site, and even serious complications such as vascular injury, nerve injury, and deep infection [3]. In addition, there are limits to the size, shape, and quantity of autologous bone that can be harvested for grafting. In addition, there are differences in the quality of autologous bone among individuals and age groups [6, 7]. For instance, the elderly generally have poor bone for grafting while patients with nonunion may have genetic factors that prevent bone healing at the donor site as well as the primary fracture site [6].

Bone morphogenetic proteins constitute a family of soluble bone matrix glycoproteins that induce migration, proliferation, and differentiation of undifferentiated mesenchymal stem cells to form osteoblasts and chondroblasts. These differentiated cells then synthesize collagen to form calcified bone tissue, promoting bone tissue repair and angiogenesis [9]. Past studies have shown that BMPs not only promote nonunion healing, but also reduce infection and pain [7, 12, 13, 16, 27, 28]. In fact, healing rates of over 90% have been reported in nonunion cases using BMP treatment [11, 13]. However, several studies have concluded that combining BMP with bone transplantation does not improve outcome and only increases the cost of treatment [29, 30]. For instance, Hackl et al. [23]. concluded that autologous bone grafting alone is equally effective and less costly than combined recombinant BMP and autologous bone grafting for aseptic nonunion of the humerus, femur, or tibia. Others have speculated that the development of BMP treatment may be driven largely by potential profits rather than improved efficacy and safety given the huge market potential of bone graft substitutes [24, 26, 30]. Previous studies on BMP efficacy are difficult to compare because of the differences in the study design, inclusion criteria, and types of nonunion. Only two meta-analyses have evaluated BMP for nonunion patients, with discrepant conclusions. Schenker et al. found a faster healing rate in the BMP treatment group, while Dai et al. [14] found no significant difference in healing rate, secondary surgery rate, or infection rate between the BMP and control groups. However, these conclusions were limited by the small sample sizes and poor quality of the included studies.

The results of this meta-analysis are that (1) BMP does not significantly improve the final extent of healing; (2) addition of BMP to autologous bone transplantation reduces fracture healing time, although treatment cost is higher; (3) BMP alone can reduce operation time and intraoperative blood loss; (4) addition of BMP improves postoperative function; and (5) addition of BMP does not influence the infection rate or rate of secondary surgery. The study by Yin et al. [22] found no increase in operation time when adding BMP treatment during bone grafting. However, most of the studies did not provide specific descriptions of the operation time and procedure, so the effect of adding BMP treatment is still uncertain.

It has been reported that the bone induction effect of BMP is not superior to autologous bone transplantation [16, 21, 31] and that BMP actually results in slower bone healing rate than autologous bone grafting alone (although the difference was not statistically significant). However, a multitude of factors ultimately contribute to the outcome, and different conditions require specific treatments, all of which may obscure the benefits of BMP. Nonetheless, BMP treatment was found to benefit certain outcome variables in this meta-analysis, suggesting BMP as a viable alternative or safe adjuvant for autologous bone grafts. Due to high cost, however, early studies did not recommend BMPs as a routine treatment for bone non-attachment. In contrast, recent cost-effectiveness studies support the use of BMPs in the treatment of persistent nonunion [30, 32–34]. Early use of BMPs may be a cost-effective strategy for treating severe cases of bone and soft tissue damage given the costs of prolonged hospitalization, medication, repeated surgical failure, and disability [30, 32–34].

The following limitations of this meta-analysis should be acknowledged. First, the pooled sample included non-randomized controlled studies, some of which did not specify group allocation or blinding, thereby introducing a risk of bias. Second, many of the studies were of small sample size. Third, long bone nonunion most often occurs in the tibia, and more than half of the cases included in the sample were patients with tibial nonunion. Therefore, the relevance of our conclusions to other long bones is less certain. Fourth, some of the studies did not specifically describe the follow-up time, so some postoperative complications and secondary operations may not have been reported. Fifth, many independent variables can affect fracture nonunion (e.g., fracture type, mechanical fixation, amount and mode of autologous bone transplantation, dose and type of BMP). Additional multicenter randomized studies are needed to control for preexisting factors associated with fracture nonunion.

In conclusion, BMP alone can improve postoperative function, shorten operation time, and reduce intraoperative blood loss in cases of long bone nonunion. Therefore, BMP may reduce done-site complications from bone extraction and provide a new treatment option for patients with poor donor bone quality or poor surgical tolerance. Bone morphogenetic protein combined with autologous bone transplantation also appears to accelerate fracture healing. However, the current evidence does not support the widespread promotion and application of BMP for improved outcomes. Large-scale clinical studies are still needed to comprehensively analyze its efficacy and economic benefits.

## Data Availability

The datasets generated during and/or analyzed during the current study are available from the corresponding author on reasonable request.

## Abbreviations

BMP: Bone morphogenetic protein
CNKI: China Biomedical Literature Database
NOS: Newcastle-Ottawa Scale
WMD: Weighted mean difference
RR: Risk ratio
RCT: Randomized controlled trial
CI: Confidence interval
